# Metabolic Analysis of Potential Key Genes Associated with Systemic Lupus Erythematosus Using Liquid Chromatography-Mass Spectrometry

**DOI:** 10.1155/2021/5799348

**Published:** 2021-10-04

**Authors:** Li Zeng, Nian Chen, Junlin Liao, Xu Shen, Shenghua Song, Feng Wang

**Affiliations:** Department of Medical Cosmetology, The First Affiliated Hospital, Hengyang Medical School, University of South China, Hengyang, Hunan 421001, China

## Abstract

The biological mechanism underlying the pathogenesis of systemic lupus erythematosus (SLE) remains unclear. In this study, we found 21 proteins upregulated and 38 proteins downregulated by SLE relative to normal protein metabolism in our samples using liquid chromatography-mass spectrometry. By PPI network analysis, we identified 9 key proteins of SLE, including AHSG, VWF, IGF1, ORM2, ORM1, SERPINA1, IGF2, IGFBP3, and LEP. In addition, we identified 4569 differentially expressed metabolites in SLE sera, including 1145 reduced metabolites and 3424 induced metabolites. Bioinformatics analysis showed that protein alterations in SLE were associated with modulation of multiple immune pathways, TP53 signaling, and AMPK signaling. In addition, we found altered metabolites associated with valine, leucine, and isoleucine biosynthesis; one carbon pool by folate; tyrosine metabolism; arginine and proline metabolism; glycine, serine, and threonine metabolism; limonene and pinene degradation; tryptophan metabolism; caffeine metabolism; vitamin B6 metabolism. We also constructed differently expressed protein-metabolite network to reveal the interaction among differently expressed proteins and metabolites in SLE. A total of 481 proteins and 327 metabolites were included in this network. Although the role of altered metabolites and proteins in the diagnosis and therapy of SLE needs to be further investigated, the present study may provide new insights into the role of metabolites in SLE.

## 1. Background

Systemic lupus erythematosus (SLE) is an autoimmune disease, which is related to substantial morbidity and increased mortality [1]. The incidence rate of SLE in China is about 50-60/100000 and is higher in women than in men [2]. Dysregulation of a number of innate immune pathways has been implicated in the pathogenesis of SLE [3, 4]. For example, disturbance of interferon-*α* (IFN-*α*) homeostasis is crucial to the pathogenesis of SLE [5]. Enhanced T cell antigen receptor (TCR) signaling and immune complexes (IC) are also reported to be related to SLE [6]. Moreover, the important role of TNF alpha in the autoimmune diseases such as SLE is widely accepted [7]. The biological mechanism underlying the development of SLE remains unclear. Therefore, it is of great significance to understand the mechanisms of the development of SLE and provide new strategies for the effective therapy for SLE.

Autoantibodies are one of the hallmarks of SLE, whose overproduction led to the clinical manifestations of SLE [8]. Antinuclear antibody (ANA) is the most commonly used biomarker of SLE, whose sensitivity is high but specificity is low; due to that, it could also be detected in other autoimmune diseases [9]. Thus, we need to identify new SLE biomarkers with higher sensitivity and specificity.

Metabolomics is a technology that is widely used to identify disease biomarkers and provide detailed information on disease progression because metabolites are the end products of DNA, RNA, and proteins [10]. Metabolomic variants represent an interaction of genetic and environmental factors and are associated with disease states, which could provide new insight into the progression of disease [11]. Metabolomics has been successfully used to define the metabolic features of multiple human diseases [11]. For example, Guo et al. identified a series of potential biomarkers for the diagnosis of fatty liver hemorrhagic syndrome by serum metabolic profiling [12]. Chen et al. reported blocked tricarboxylic acid (TCA) cyclic metabolism plays an important role in chronic DILI-associated cirrhosis [13]. Zhang et al. identified 11 metabolites, such as hexadecanoic acid (C16:0), as potential serum biomarkers for diabetic kidney disease [14]. As a high-throughput method, metabolomics could detect thousands of serum metabolites once during the different progression stages of human diseases, which is suitable for biomarker discovery. Very interestingly, several recent studies also demonstrated this finding in SLE. For example, Leda et al. reported serum metabolomic signatures can predict subclinical atherosclerosis in patients with SLE. George et al. found increased apolipoprotein-B : A1 ratio predicts cardiometabolic risk in patients with juvenile-onset SLE. However, the roles of metabolomics in SLE remained to be unclear. In this study, we identified altered proteins and metabolites in SLE by applying an untargeted metabolomic analysis with UPLC-Q-TOF/MS. The identification of a series of novel proteins and metabolites may provide novel biomarkers for SLE.

## 2. Materials and Method

### 2.1. Sample Preparation

Samples were thawed at 4°C, and 100 *μ*L blood serum per sample was transferred to a new tube and then added 400 *μ*L methanol (MeOH) and 400 *μ*L acetonitrile. After vortexing 30 s and sonicating 10 min, proteins were prone to precipitate by being incubated 1 h at 20°C. After centrifugation, the supernatant was dried in a vacuum concentrator. The extracts were then resuspended in 100 *μ*L of 1 : 1 acetonitrile : H_2_O and sonicated 10 min and stored at -80°C.

### 2.2. Liquid Chromatography-Mass Spectrometry (LC-MS)/MS

The supernatant was analyzed by HPLC-MS/MS on TripleTOF™ 6600plus mass spectrometer (AB SCIEX, USA), coupled to an Agilent 1290 liquid chromatography system (Agilent, USA). For LC separation, the ACQUITY UPLC, BEH C18 column was used. 5 *μ*L sample was injected and separated with a 12 min gradient. The electrospray ionization mass spectra were acquired in positive and negative ion mode, respectively. The ion spray voltage was set to 5000 V for positive mode and 4000 V for negative mode.

### 2.3. Data Processing

ProteoWizard (version 3. 0. 6150) was used for normalizing [15]. All of MS files (mzXML format) were processed using R package “XCMS” (version 1.46.0) for peak detection and alignment [16]. Metabolite identification was achieved by MetDNA (http://metdna.zhulab.cn/), with the MS1 peak table and MS2 data files (mgf format). In order to select differential metabolites, the MS1 peak table was uploaded to MetaboAnalyst (https://www.metaboanalyst.ca) to perform differential metabolite discovery [17]. Principal component analysis (PCA) and partial least squares discriminant analysis (PLS-DA) were performed using normalized peak table by total intensity to investigate a possible separation of metabolite profiles between control and MG samples, and fold changes and *p* values (assessed by the Student *t*-test) were computed. The discovery data set contained 76533 features, and 4569 features were significantly differentiated with fold changes greater than 1.5, *p* value less than 0.05, and VIP greater than 1.5.

### 2.4. Enrichment Analysis

Enrichment analysis was performed using the Database for Annotation, Visualization, and Integrated Discovery (DAVID) v6.8 (https://david.ncifcrf.gov/) [18].

### 2.5. Protein-Protein Interaction (PPI) Network Analysis

We used STRING (https://string-db.org/) [19] to construct the PPI network in SLE.

### 2.6. Statistical Analysis

The data were analyzed by SPSS 22.0 software. Student's *t*-test was used where appropriate. A *p* value less than 0.05 was considered as statistically significant.

## 3. Result

### 3.1. Identification of Altered Proteins in SLE

In the present study, 3 SLE samples and 3 healthy control samples were used to identify SLE-related proteins. The SDS-PAGE results show that the protein quality of each sample is good, the total amount of each sample is sufficient, and the parallelism between samples is good (Figure 1(a)). Base peak analysis showed relative abundance of peaks eluting at different times is relative abundance (Figure 1(b)).

After normalizing the raw data in the limma package [20] using corrected *p* value < 0.05 of R software, we revealed 21 proteins were induced and 38 reduced proteins in SLE compared to normal samples. The top 5 induced proteins included ORM1, ORM2, APOC3, APOC4, and IGLV3-10. The top 5 reduced proteins included THBS4, APEH, CBLN4, KIT, and OMD. The top 10 upregulated and 10 downregulated proteins in SLE are listed in Table 1. The heat map (Figure 1(c)) and volcano map (Figure 1(d)) of all DEGs are shown in Figure 1. PCA revealed the SLE samples were clustered and separated from normal samples (Figure 1(e)).

### 3.2. Functional Enrichment Analysis of Altered Proteins in SLE

To explore the potential function of the proteins with altered levels in SLE, we performed GO and KEGG pathway analysis. Our results showed that these proteins were related to regulate platelet degranulation, bone mineralization involved in bone maturation, activated T cell proliferation, cell division, acute-phase response, multicellular organism reproduction, ovulation from ovarian follicle, regulation of gene expression by genetic imprinting, and glycolate metabolic process (Figure 2(a)). For CC enrichment, these proteins were mainly related to insulin-like growth factor ternary complex, platelet dense granule lumen, exocytic vesicle, nucleosome, platelet dense tubular network, and protein C inhibitor complex (Figure 2(a)). For MF enrichment, these proteins were mainly related to protease binding, dipeptidyl-peptidase activity, heparin binding, and metalloendopeptidase activity (Figure 2(a)).

The domain enrichment analysis showed proteins with altered levels in SLE were related to peptidase S9, serine active site, peptidase S9, prolyl oligopeptidase, catalytic domain, alpha-1-acid glycoprotein, coiled-coil domain, IlGF, insulin, conserved site, insulin-like superfamily, insulin family, insulin-like, and insulin-like growth factor (Figure 2(b)). KEGG enrichment analysis showed proteins with altered levels in SLE were related to growth hormone synthesis, secretion and action, AMPK signaling pathway, and p53 signaling pathway (Figure 2(c)). The protein location analysis showed these proteins mainly located in extracellular, endoplasmic reticulum, plasma membrane, mitochondria, cytosol, nucleus, and peroxisome (Figure 2(d)).

### 3.3. PPI Network Establishment

To reveal the potential relationships among proteins with altered levels in SLE, a PPI network was built using the STRING database. 43 nodes and 111 edges were included in the PPI network (Figure 3). Based on network analysis, we identified 9 hub proteins with degree > 10, including alpha 2-HS glycoprotein (AHSG), insulin-like growth factor 1 (IGF1), orosomucoid 2 (ORM2), von Willebrand factor (VWF), orosomucoid 1 (ORM1), serpin family A member 1 (SERPINA1), insulin-like growth factor 2 (IGF2), insulin-like growth factor binding protein 3 (IGFBP3), and leptin (LEP). These hub proteins connected with more 10 other proteins.

### 3.4. PCA of Serum Samples in SLEs

As presented in Figure 4, PLS-DA plots were applied to characterize the metabolic profiles for both positive (Figures 4(a) and 4(b)) and negative (Figures 4(c) and 4(d)) modes. We revealed SLEs compared to controls showed distinct separations in the score plots, indicating global changes to serum metabolite composition in SLE.

### 3.5. Altered Metabolites Were Identified in SLE

Furthermore, altered metabolites were identified in SLE. In positive modes, 3405 significant altered metabolites were identified, including 3289 induced metabolites and 117 reduced metabolites (Figures 5(a) and 5(c)). In negative modes, 1165 significant altered metabolites were identified, including 136 induced metabolites and 1028 reduced metabolites (Figures 5(b) and 5(d)). Also, the correlation among these differentially expressed metabolites was also analyzed (Figures 5(e) and 5(f)).

By merging both the positive and negative modes, we identified 4569 differentially expressed metabolites in SLE serum samples, including 1145 reduced metabolites and 3424 induced metabolites in SLE samples compared to normal samples. The most differently expressed metabolites included phoenicoxanthin, L-(+)-anaferine, isorenieratene, psilocin, (S)-reticuline, deoxytubulosine, tetrahomomethionine, cellopentaose, lobeline, 2-hexaprenyl-6-methoxy-1,4-benzoquinone, nebramycin 5′, octacis-undecaprenol, glycochenodeoxycholate 7-sulfate, coumaryl acetate, S-[2-(N7-guanyl)ethyl]-N-acetyl-L-cysteine, protodeoxyviolaceinic acid, and catharanthine (Figure 5).

### 3.6. Pathway Enrichment Analysis of Altered Metabolites

Pathway enrichment was performed using MetaboAnalyst 4.0, and the results are showed in Figure 6. The altered metabolites are related to valine, leucine, and isoleucine biosynthesis; one carbon pool by folate; tyrosine metabolism; arginine and proline metabolism; glycine, serine, and threonine metabolism; limonene and pinene degradation; tryptophan metabolism; caffeine metabolism; and vitamin B6 metabolism (Figures 6(a) and 6(b)).

### 3.7. Construction of Differently Expressed Protein-Metabolite Networks

We next constructed differently expressed protein-metabolite network to reveal the interaction among differently expressed proteins and metabolites in SLE. As shown in Figures 7 and 8, 481 proteins and 327 metabolites were included in this network.

## 4. Discussion

Over the past few decades, a number of regulatory factors related to the progression of SLE have been identified. For example, targeting Kv1.3 channels in T lymphocytes can correct disease manifestations associated with SLE [21]. Systemic lupus erythematosus favors the production of double-negative T cells that produce IL-17 [22]. The REDD1/autophagy pathway is mediated by tissue factor (TF) and interleukin-17a (IL-17a) promotes thrombotic inflammation and fibrosis in human SLE [23]. NF-*κ*B inducible kinase is a therapeutic target for SLE. It should be noted that some previous studies have identified multiple central regulators of SLE, such as Zhang et al. who identified 23 different metabolites and 5 interference pathways between the two groups through fecal metabolomic analysis, including aminoacyl-tRNA biosynthesis [24]. Kalantari et al. identified alanine, 2,2-dimethylsuccinic acid, and 3,4-dihydroxyphenylacetaldehyde as diagnostic criteria for lupus nephritis [25]. Yan et al. profiled the fecal metabolome using gas chromatography-mass spectrometry and explored the potential roles of metabolites in the diagnosis and progression of SLE [26]. In the present study, we revealed 21 proteins were induced and 38 reduced proteins in SLE compared to normal samples with UPLC-Q-TOF/MS.

In addition, we performed bioinformatics analysis of altered proteins in SLE patients. Our findings indicated altered proteins are involved in multiple immune pathways, such as platelet degranulation, upregulation of activated T cell proliferation, cell division, acute phase response, and glycolate metabolism. Our research suggests that the immune pathway plays an important role in SLE. Analysis of KEGG pathway showed that TP53 and AMPK signals were related to SLE. Of note, our findings were consistent with previous report that T cell proliferation had a key role in SLE, which was also considered as a fundamental immunologic characteristic of SLE. In this study, we found that AHSG, VWF, IGF1, ORM2, ORM1, SERPINA1, IGF2, IGFBP3, and LEP were closely related to SLE and played a crucial role in the occurrence and development of SLE. AHSG is a glycoprotein synthesized by a variety of fetal tissues. It has been shown that in SLE patients, the level of AHSG is reduced and is inversely associated with carotid intima-media thickness, which is consistent with our findings, suggesting that AHSG is a biomarker of atherosclerosis and can be used to evaluate SLE progression [27, 28]. IGF1 activates the cell proliferation pathway and inhibits cell apoptosis, which is involved in tumor growth and is required for B cell-independent T cell activation, the hallmark of SLE. Free IGF1 has a positive metabolic role in SLE, which may indirectly inhibit cellular immune response by suppressing B cell and T cell activity [29]. Serum IGFBP-3 was higher in systemic sclerosis than in controls, and elevated IGFBP-3 levels were related to a lower incidence of telangiectasia in systemic sclerosis [30]. Leptin is a cytokine-like hormone, which can control energy consumption. Leptin had a key role in immune imbalance in SLE. Multiple reports revealed elevated leptin levels promote SLE progression by inducing autoantibody production and inhibiting immune regulation. Leptin induced the Th17 differentiation by activating NLRP3 inflammatory bodies [31]. In humans, the hominoid bone meal (ORM) family contains two genes, ORM1 and ORM2. The ORM family contains three subtypes, ORM1, ORM2, and ORM3, which are the acute phase proteins of inflammatory response [32]. Our study is the first to show that ORM1 and ORM2 are associated with SLE.

By comparing the metabolism of SLE patients with that of controls, we identified a series of metabolites, including phoenicoxanthin, L-(+)-anaferine, isorenieratene, psilocybin, (S)-reticuline, deoxyuracil, tetramethionine, cellopentaose, 2,3-bis-(O-phytyl)-sn-glycero-1-phospho-L-serine, lobeline, 2-hexenyl-6-methoxy-1, 4-benzoquinone, and nebramycin 5′. Bioinformatics analysis showed that the elevated levels of these metabolites were associated with biosynthesis of valine, leucine, and isoleucine; tyrosine metabolism; tryptophan metabolism; and vitamin B6 metabolism. Interestingly, these metabolisms are associated with SLE. For example, vitamin B6 was inversely associated with unchanged/increased glucocorticoid dose, suggesting that vitamin B6 may prevent GC dose increase. A prospective study of Japanese women found an inverse association between vitamin B6 intake and risk of active disease. Degradation of tryptophan is found in patients with SLE. Mood disorder in SLE is caused by decreased serum and brain tryptophan and antiribosomal P protein antibodies [33]. Dysregulation of the gut microbiota and altered tryptophan catabolism lead to autoimmunity in lupus-prone mice in a mouse model. Our results and previous reports suggest that tryptophan deficiency and vitamin B6 may be associated with neurological/psychiatric disorders in SLE.

Several limitations should also be noted. First, only 3 SLE samples and 3 healthy controls were used to identify altered proteins in SLE. The sample size is limited. More clinical samples will be collected for further confirmation. Second, many metabolites were identified to be related to SLE. However, the roles of these metabolites in SLE remained to be further confirmed.

Altogether, we identified 21 proteins that were upregulated by SLE and 38 that were downregulated. By PPI network analysis, we identified 9 central genes of SLE, including AHSG, VWF, IGF1, ORM2, ORM1, SERPINA1, IGF2, IGFBP3, and LEP. In addition, we identified 4569 metabolites differentially expressed between SLE serum samples and normal samples, including 3le reduced metabolites and 3424 induced metabolites. Bioinformatics analysis showed that the protein changes of SLE were related to the regulation of multiple immune pathways, TP53 signaling, and AMPK signaling. In addition, we found that these altered metabolites are involved in amino acid metabolism and vitamin B6 metabolism. Although the exact role of these metabolites in the diagnosis and treatment of SLE disease requires further investigation, this study may still provide novel information to understand the role of metabolites in SLE.

## Figures and Tables

**Figure 1:** Identification of altered proteins in SLE. (a) The SDS-PAGE results show the protein quality of each sample. (b) Base peak analysis showed relative abundance of peaks eluting at different times. (c) Heat map analysis of altered proteins in SLE. (d) Volcano map analysis of altered proteins in SLE. (e) The PCA score plots of serum samples from SLE patients and control patients.

**Figure 2:** Functional enrichment analysis of altered proteins in SLE. (a) GO analysis of altered proteins in SLE. (b) The domain enrichment analysis of altered proteins in SLE. (c) KEGG analysis of altered proteins in SLE. (d) The protein location analysis of altered proteins in SLE.

**Figure 3:** PPI network analysis of altered proteins in SLE.

**Figure 4:** PLS-DA analysis for SLE and control samples. (a, b) PLS-DA plots for SLE versus control separation in positive mode with 2D and 3D format. (c, d) PLS-DA plots for SLE versus control separation in negative mode with 2D and 3D format.

**Figure 5:** Differentially expressed metabolites were identified in SLE. Volcano map analysis of altered metabolites in SLE in (a) negative mode and (b) positive mode. Volcano map analysis of altered metabolites in SLE in (c) negative mode and (d) positive mode. Correlation analysis of altered metabolites in SLE in (e) negative mode and (f) positive mode.

**Figure 6:** (a, b) Pathway analysis of significant altered metabolites in SLE.

**Figure 7:** Construction of differently expressed protein-metabolite networks—1. The figure shows the relationship between compounds, enzymes, reactions, and proteins. Different shapes represent different molecular types: hexagons represent compounds; diamonds represent reactions; circles represent genes; rectangles represent enzymes. The connection between them indicates their relationship.

**Figure 8:** Construction of differently expressed protein-metabolite networks—2. The figure shows the relationship between compounds, enzymes, reactions, and proteins. Different shapes represent different molecular types: hexagons represent compounds; diamonds represent reactions; circles represent genes; rectangles represent enzymes. The connection between them indicates their relationship.

**Table 1:** The top 10 upregulated and 10 downregulated proteins in SLE are listed.

Gene name	Abundances SLE1	Abundances SLE2	Abundances SLE3	Abundances CON1	Abundances CON2	Abundances CON3	Regulation	SLE/CON	*p* value
ORM1	192.3	163.1	135.6	34	37.6	37.5	Up	4.500	0.001
ORM2	176	147.8	146.7	41.9	45.8	41.8	Up	3.633	0.000
APOC3	167.6	141.7	119.2	56.9	58.7	55.9	Up	2.499	0.004
APOC4	134.8	99.4	179.2	59.1	64.5	63	Up	2.215	0.031
IGLV3-10	153.3	94.1	142.4	78.6	64	67.5	Up	1.855	0.033
MMP3	124.4	143.1	111.2	80.6	72.1	68.6	Up	1.711	0.006
SAA4	117.4	117.5	134	77.8	81	72.3	Up	1.596	0.002
IGLV3-27	131.4	112.7	115.5	74.9	68	97.5	Up	1.496	0.020
VWF	133.5	116.2	109	78	83.1	80.3	Up	1.486	0.006
PIGR	105.2	111.1	140.3	81.5	88.1	73.8	Up	1.465	0.031
LUM	73.9	89.6	79.6	107.1	121.4	128.6	Down	0.681	0.008
PI16	67.3	98.5	76.8	106.2	122.2	129	Down	0.679	0.029
AHSP	82.7	69	89.6	136.6	95.5	126.6	Down	0.673	0.047
IGF2	81.5	77.4	79.2	117.4	126.4	118.1	Down	0.658	0.000
FAP	83.3	70.3	79.7	116.7	127.1	123	Down	0.636	0.001
THBS4	74	74	79.7	115.6	126.1	130.5	Down	0.612	0.001
APEH	77.3	71.3	78.4	118.8	99.6	154.6	Down	0.609	0.040
CBLN4	71.8	78.9	75.7	98.8	140	134.9	Down	0.606	0.020
KIT	71.2	77.6	77.4	135.8	123.2	114.8	Down	0.605	0.002
OMD	82.4	69.6	70.1	105.3	119.5	153.1	Down	0.588	0.025

## Data Availability

The data used in this study are included within the article. The data and materials in the present study are available from the corresponding author on reasonable request.
